# Sex Moderated Mediation of the Musculoskeletal Fitness in Relationship between High-Intensive Interval Training Performing during Physical Education Classes and Cardiorespiratory Fitness in Healthy Boys and Girls

**DOI:** 10.1155/2022/8760620

**Published:** 2022-01-17

**Authors:** Jarosław Domaradzki, Dawid Koźlenia, Marek Popowczak

**Affiliations:** ^1^Faculty of Physical Education and Sport, Biostructure Unit, University School of Physical Education, Wroclaw, Poland; ^2^Faculty of Physical Education and Sport, Department of Team Sports Games, University School of Physical Education, Wroclaw, Poland

## Abstract

High-intensive interval training (HIIT) is indicated as a means of improving cardiorespiratory fitness (CRF) and musculoskeletal fitness (MSF). The relationship between CRF and MSF was examined too. Little is known about gaining CRF from HIIT independence of MSF in adolescents. Therefore, this study is aimed at investigating whether MSF mediated the relationship between HIIT and CRF and whether sex moderate this relation. The study sample included 122 individuals (45 boys, 77 girls) 16.12 ± 0.38 years of secondary school age. Participants were assigned to the HIIT intervention or control groups. The intervention lasted 14 minutes during one physical education lesson per week for ten weeks. Outcome and potential mediator were residual changes calculated from pre- and postintervention results of MSF components: handgrip (HG), sit-ups (ABS), sit-and-reach (FL), vertical jump (VJ), and Harvard step-test representing cardiorespiratory fitness (CRF). MSF index (MSFI) was calculated as a construct, agglomerating all MSF, and tested its usefulness. HIIT significantly impacted CRF in boys and girls (*B* = 2.32, *p* = 0.032; *B* = 2.28, *p* = 0.005, respectively). The impact of the HIIT program on the ABS and FL was observed only in girls. The moderation effect of sex was confirmed. Significant effect of HIIT on CRF decreased (*B*_direct_ < *B*_total_) and was no significant after including FL (*B* = 1.46, *p* = 0.62)—complete mediation, but no ABS (*B* = 2.97, *p* = 0.001)—partial mediation. CRF was mediated by changes in ABS (*B* = 2.28, *p* < 0.001) and FL (4.18, *p* < 0.001). MSFI was not mediating; its usefulness was limited. HIIT is an effective tool in the development of CRF in both sexes. MSF played a limited role in the relationship between HIIT and CRF. It suggested different mechanisms in both sexes: girls who performed better to the HIIT had better values of FL and ABS, but not boys. HIIT intervention involved modifications in ABS or FL, which also influenced the increase of CRF.

## 1. Introduction

Physical fitness (PF) is a construct that contains several components usually separated into cardiorespiratory fitness (CRF) and muscular fitness (MF) [1]. In the Health-Related Fitness (H-RF) concept, MF is linked to flexibility and builds together a multidimensional construct—musculoskeletal fitness (MSF) [2, 3]. Studies on MSF are based mainly on these components: muscle strength (static and dynamic) and flexibility [4–6]. Less often, global, agglomerated indexes were created and investigated. As an H-RF component [7–9], MSF is considered a health marker [10, 11]. Each MSF item can predict health status in childhood or adolescence and later life phases [3, 10].

Cardiorespiratory fitness (CRF) is the body's circulatory and respiratory systems' ability to supply fuel and oxygen during sustained physical activity [12]. CRF reflects the power of the lungs, blood, heart, and muscles to transport and utilize O_2_ via the aerobic metabolic pathways, thus determining a person's level of CRF has both general and clinical applications [13].

Actions taken to address the problem of low CRF and MSF include developing programs for promoting physical activity and their implementation in physical education (PE) in schools. Primary and secondary schools are ideal places to implement different interventions and physical activity programs [14]. More than 90% of children worldwide attend primary school [15]. Therefore, physical education classes are considered an ideal setting to promote healthy physical activity [16]. Physical education classes can create natural conditions for participation in PA due to the regularity of lessons and the possibility of controlling the volume and intensity of physical effort what an effective strategy to improve health status [17]. It is a crucial issue nowadays of the COVID-19 pandemic during lockdowns that physical activity decreases significantly among adolescents [18].

Some scientific results showed that HIIT during physical education classes could be highly effective for cardiorespiratory status improvement among normal and overweight adolescents [19]. The same research indicates that short intensive training intervention could be as effective as prolonged PE and saving time. HIIT improves endurance and decreases body fat. The effects of HIIT programs on CRF and MSF were widely described [19–24]. On the other hand, several studies established the relationships between CRF (and its marker—maximal oxygen uptake) and MSF [25–28]. Generally, the HIIT method improves adolescents' maximal oxygen uptake related to CRF and morphological features (WHR, BMI, MFR) related to MSF and decreased disease biomarkers, as lower BMI [22, 24].

However, according to our knowledge, there is a lack of studies that have examined interrelationships among HIIT, MSF, and CRF in adolescents. Youth are an essential target population because of the final stage of maturation which is critical for growth. It is manifested, on the one hand, by an increase in an unwillingness to physical activity and, on the other hand, by greater susceptibility to the unhealthy effects of physical inactivity (increased body fat, BMI, WHR indices, and risk factors for metabolic syndrome) [29, 30].

A clear understanding of HIIT associations with MSF and CRF is crucial for identifying areas to target interventions. The potential mediating effect of MSF in relationships between HIIT and CRF is likely and plausible, as HIIT affects MSF, as indicated above [19–28, 31]. These findings suggest a mediating effect of MSF on the relationships between HIIT and CRF. Thus, the main question is whether the HIIT program partially produces the observed outcomes in CRF via changes in MSF (mediator variable). Therefore, the main aim of the present study was to examine whether MSF mediated the associations of HIIT and CRF in adolescents. Specifically, we aimed to (1) examine the impact of HIIT on CRF, (2) determine whether each component of MSF (single test's results), as well as MSFI (composite construct), mediate effects of HIIT on CRF, and (3) specify whether the sex is moderating variable when mediation by MSF is present. Modeling relationships was based on Baron and Kenny [32] procedure.

## 2. Material and Methods

The methods were described in detail and summarized in our previous study [33].

### 2.1. Ethics

The Senate Research Ethics Committee approved the University of Physical Education research in Wrocław (Poland) following human experiments' institutional ethical requirements under the Helsinki Declaration (consent number: ECUPE no: 19/2019). All students and their legal guardians were informed in detail about the study's design, including the potential risks and benefits, before providing their written informed consent to participate. Then, all legal guardians were asked to write a consent document before testing. The surveys were conducted by faculty and staff of the University of Physical Education in Wrocław in cooperation with teachers at school.

### 2.2. Power Calculation

Before recruitment, a power calculation was conducted to determine the required sample size to detect medium-sized mediation effects [34]. Based on 80% total power, a-path and b-path (two arms of indirect impact, through mediator) equal 0.8944, an *α* level of 0.05, and minimum effect size of 0.05–0.10, it was calculated that 81–159 participants would be required to detect a between-group difference in outcome values. To calculate the sample size, G∗Power tool (Sydenham Institute of Management Studies and Research and Entrepreneurship Education) was used [35].

### 2.3. Participants

In this study, participants comprised 122 healthy individuals, 16 years of age (16.12 years ± 0.38), BMI normal range, and blood pressure norm (normotensive systole and diastole). Adolescents studied in a Polish comprehensive secondary school and lived in a big city (about 650,000 inhabitants). The sex distribution was 45 males and 77 females. Concerning the sex distribution, although there is a marked, slight bias towards the female group, this proportion represents the population in the field of studies analyzed.

### 2.4. Procedure

An intervention group (IG) (*N* = 64, boys: 27, girls: 37) and a control group (CG) (*N* = 58, boys: 18, girls: 40) were randomly selected from all first-year secondary students (six classes total) in the school before the school year began. The inclusion criteria were normal BMI and normotensive blood pressure.

In short, the tests most adequate to measure functional traits and motor abilities were used in this study. All the tests were conducted one day, from 8 : 00 a.m. to 1 : 00 p.m., in sports halls in the same conditions for each group. Each participant wore a T-shirt, shorts, and shoes. Only anthropometric measurements were conducted without shoes.

Measures were taken pre- and postintervention in the following order: anthropometric measurements, muscular strength and flexibility, power of legs, and cardiovascular fitness. Each measurement's protocol was based on HR-F measurement recommendations.

### 2.5. Intervention

Participants included in IG performed a 14-minute HIIT exercise regimen based on a Tabata Training Program (TAP), presented as a video during one of three weekly physical education class lessons carried out in the fitness room. The TAP was used in the experimental group (EG) for ten weeks (from the 5th week of the school year) from 9 : 00 a.m. to 12 : 30 p.m. The remaining physical education class lessons were conducted according to the school's standard curriculum for first-year secondary students. CG participants followed the physical education class curriculum without any interval training exercises. Participants were instructed to maintain normal activity levels and refrain from other organized physical activity except for physical education classes [36]. During the other two physical education classes in the week, activities included various team sports, dance, and gym exercises.

### 2.6. Anthropometric Measurements

Two height measurements were made with an accuracy of 0.1 cm using anthropometers (GPM Anthropological Instruments). Bodyweight was measured with a body composition—InBody230 (InBody Co. Ltd., Cerritos, CA, USA). The above data were used to calculate BMI. No bioelectric impedance results were studied in this work.

### 2.7. Cardiorespiratory Fitness

The physical fitness index (FI) that defines cardiovascular fitness (CRF) was determined using the Harvard step-test [37]. Many studies used the Harvard step-test as a method used to access CRF developed by Brouha et al. [38]. In the Harvard step-test, oxygen consumption is usually estimated from equations. The validity of the Harvard step-test to predict VO_2max_ was proved very quickly after introducing in physiological measurements in many studies [38–40]. Correlations between direct and predicted VO_2max_ were calculated as *r* = 0.618-0.805, and the repeatability was acceptable (ICC = 0.63) [41]. In the Harvard step-test, participants stepped up and down on a 16.25-inch (41.3 cm) high stool at a pace of 30 cycles per minute with a metronome set at 120 bpm. The exercise continued for up to 300 seconds, less if participants became fatigued. Recovery pulse was recorded within 1.5 minutes of recovery. Before each test, Polar H1 heart rate monitors were fitted to each student as per the above process. Resting heart rate and its changes during exercise and recovery pulse were measured. Heart rate monitors sampled participants' pulse at 5-second intervals and were transmitted to a smartwatch (Polar, Polar Electro; Kempele, Finland). FI was calculated using the following formula [42]: FI = (100 × *L*)/(5.5 × *p*), where *L* is the duration of the test in seconds, *L* < 300 seconds, and *p* is the heart rate within 1.5 minutes after the subject stopped the test.

### 2.8. Musculoskeletal Fitness

To determine the musculoskeletal fitness components, the following tests were conducted: hand muscular static strength measurement (HG) and hand dynamometer (Baseline, FEI, Irvington, NY, USA) were used; 30-second sit-up test (abdomen muscular strength (ABS)); sit-and-reach test (flexibility (FL)); vertical jumping ability (power of muscles of leg power (VJ)) and jumps were performed on a g-force tracker (Vert Jump; VERT, Fort Lauderdale, USA). All tests demonstrated very good test-retest reliability and validity [43]. The measures mentioned above were used previously by other authors in studies among adolescents [42, 44, 45].

### 2.9. Statistical Analysis

The Shapiro-Wilk test was used to evaluate the normality of data distribution, and all variables showed a normal distribution. Descriptive statistics of anthropometric features were presented as means, standard deviations, and 95% confidence intervals (CI).

To achieve the study's purpose and solve the problem, mediation analyses were performed using the procedure described by Baron and Kenny [32] with the accompanying Jamovi's Advanced Mediation Models 1.0.4 module (Jamovie, v. 1.6, 2020). Simple regression was used to calculate the equation. The residual change was then calculated by subtracting the predicted posttest scores from the observed posttest scores, regressed on the grouping variable.

The outcome variables in mediation analysis were (1) musculoskeletal fitness index (MSFI) constructed based on the results of each motor test (HG, ABS, FL, VJ) and (2) each test itself. Thus, mediation analysis was conducted five times: composite MSF construct was evaluated independently on mediation analysis for each test. The indirect effect of composite MSF and each facet of MSF was studied to determine which motor ability as a mediator had the most significant impact on improving CRF.

All tests representing different motor components were accumulated into a joint, agglomerated index, gathering information about musculoskeletal fitness. The agglomerated MSF index was created using Multidimensional Comparative Analysis (MCA). These methods are popular in economy and econometry and used in biological studies [46]. Out of different procedures, Hellwig's pattern of development method was used. A detailed description of the steps of the process in the design of the development method was published originally by Hellwig [47].

The significance level was set at *a* = 0.05. Statistica V. 13.0 statistical package was used to analyze the study data. The accompanying Jamovi's Advanced Mediation Model 1.0.4 module (Jamovie, v. 1.6, 2020) was used to perform mediation analyses using the procedure described by Baron and Kenny [32].

## 3. Results

Table 1 presents baseline descriptive statistics of the boys' and girls' anthropometric measurements and motor tests from experimental and control groups. In addition, mean values and 95% CI of the residual changes (RC) of the outcome CRF and potential mediators (MSFI composite and HG, ABS, FL, VJ MSF's components) were presented. The analysis of residual changes was the basis for conclusions in this study.

There were not significant differences between groups at the baseline (in both sexes). However, there were significant differences in BMI between E and C groups (boys and girls) after the intervention program. Average values of BMI suggested the body mass of participants in the normal range (in all groups). There were statistically significant differences between boys and girls at the beginning of the project. Therefore, sex moderation effect on potential mediations was possible.

The effect of the HIIT on CRF was assessed based on *total effects* calculated in moderated mediation model for both sexes. Results confirmed the significant and positive impact of HIIT on CRF in the whole group (average), as well as in boys and girls, separately (average: *B* = 2.314, *p* < 0.001; boys: 2.320, *p* = 0.032; girls: *B* = 2.283, *p* = 0.005).

### 3.1. Sex Moderation Analysis

Hypothesized moderation model is presented in Figure 1. Moderation effects were represented by statistically significant interactions between categories of the moderator (sex: boys, girls) and elements of mediation model: (1) indirect effect of HIIT intervention on CRF (HIIT⇨CRF), (2) model's component: HIIT intervention on MSF (HIIT⇨MSFI, HG, ABS, FL, VJ0), and (3) model's component: MSF (MSFI, HG, ABS, FL, VJ⇨CRF). Suppose there was a significant interaction (*p* ≤ 0.05), it meant differences in the element of mediation model between both sexes. Lack of significant interaction (*p* > 0.05) meant the same effect in both sexes' elements of the mediation model.

In the first stage, interactions were investigated.  Table 2 displays *p* values for moderation effects on all three elements of the mediation model (graphically in Figure 1).

Moderation analysis revealed two MSF components that moderated mediation models: sit-ups results (ABS) and flexibility (FL). The tests significantly differentiated mediation models in both sexes. Thus, potential moderated mediation models were indicated.

In the next stage, the indirect effects were assessed to identify whether the MSF (MSFI and components) mediated the relationship between HIIT and CRF, on average and separately in boys and girls.  Table 3 displays *p* values for indirect effects.

Observed significant indirect effect in ABS and FL models in girl group suggested mediation role of these MSF's components in relationship between HIIT and FI. Neither MSFI nor HG and VJ in girls and any MSF tests in boys mediated the effects of HIIT on FI. Only models with significant indirect effects were studied in the following (3rd) stage.

### 3.2. Simple Mediation Analysis

The results from mediation analysis are shown in Table 4. As indicated previously, indirect effects in the mediation of both motor tests were statistically significant (Table 3). Overall, both MSF components in girls (ABS and FL) were positively associated with CRF. The role of ABS was lower than FL (accounted percent of mediation = 18% and 36%, respectively). It was also confirmed that HIIT affected ABS (*B* = 2.283,*p* < 0.001) and FL (*B* = 4.181,*p* < 0.001), which was manifested—more difference in pre-post ABS or FL and more difference in CRF and in HIIT participants. Furthermore, increasing differences between baseline and postintervention results were related to more gain in ABS or FL (*B* = 0.303, *p* = 0.013; *B* = 0.196, *p* = 0.013, respectively). Finally, while the indirect effects of HIIT on CRF through ABS and FL were statistically significant, the direct effect in FL was weaker and no longer significant (*B* = 1,462, *p* < 0.062). In the case of ABS, the direct effect was still significant (*B* = 2.974, *p* = 0.002). These findings indicated that FL was a complete mediator, but ABS was the partial mediator of the relationship between HIIT and FI.

## 4. Discussion

This study has to show if there is a mediation effect of MSF in HIIT impact on CFR concerning potential sex differences. Knowledge, how MSF components mediate HIIT effects on CFR could indicate how to develop MSF to improve HIIT impact on CFR and reach more benefits in CFR. Our results showed that HIIT affected CRF as well as boys and girls. However, the mediation effect was revealed throughout the flexibility and abdomen muscle strength only among girls. It showed the moderation effect of sex and the need for a deeper exploration of the MSF mediation effect among boys. The construct of MSFI usefulness was limited. However, due to potential differences between boys and girls, that index should be separated to boys and girls and consider other MSF components.

In the previous study, we confirmed the impact of the HIIT on the CFR and MSF among healthy adolescents [33]. However, now, we investigated the potential mediator—MSF components of HIIT impact on CFR. Some scientific results showed that HIIT during physical education classes could be highly effective for cardiorespiratory status improvement among normal and overweight adolescents [19]. The same research indicated that short intensive training interventions could be as effective as prolonged ones during physical education lessons, saving time. HIIT improves endurance, decreases BMI and body fat percentage, and enhances MSF [21, 23]. It showed increased muscle mass (in morphology) and muscle strength (as a functional effect) as well as cardiovascular parameters [48]. The meta-analysis evaluated school-based motor skills, and musculoskeletal fitness interventions confirmed the high effectiveness of different interval programs (HIIT with Tabata protocol) on metabolic parameters and cardiorespiratory fitness [49]. These effects were observed in our results, where boys and girls improved their CRF. Many studies show positive effects of high-intensive efforts in developing circulatory and respiratory systems. It was observed in the study by Dias et al. [50] where obese children and adolescents reached significant improvement in CFR during the HIIT program, and this effect was better in comparison to the group with continuous, moderate training. This effect is supported by improving cardiac parameters [51]. Hay et al. [52] show significant improvement in CRF with a joint decrease in body morphology parameters in 6 months. However, these effects are possible after 12 weeks of HIIT [53]. Agostinis-Sobrinho et al. [54] indicated that improving the MSF is associated with reduced cardiometabolic risk in youth. Especially, increasing muscular fitness is associated with lower blood pressure among adolescents [55]. The review by Abarzúa et al. [56] among teenagers summarizes the positive effects of HIIT on muscle and cardiovascular fitness. Moreover, this kind of physical effort seems more effective than a continuous one [57].

In the case of HIIT influence on MSF, there was significant improvement observed with better function in CRF after 12 weeks of training among adults [58]. Similar observations that are provided by Hurst et al. [59] showed higher muscular strength after HIIT, which was confirmed in a similar study by Sculthorpe et al. [60]. Brown et al. [61] showed positive effects of HIIT on CRF and MSF among young women. This effect was supported by fat mass reduction with lean muscle mass increase. Therefore, positive changes in MSF were observed by improving scores in a fitness test and VO_2max_. The HIIT effect on CRF is supported by joint development in MSF. However, due to physical fitness differences between males and females, this phenomenon could have other mechanisms between the sexes.

Abovementioned studies by Brown et al. [61] confirm HIIT results in CFR improving with joint MSF increase among females. A favorable change in body tissue could potentially cause this mediation effect. HIIT could effectively increase muscle mass among males and, therefore, drive development in MSF. Our study was revealed through ABS scores after the intervention, with combined effects in metabolic that positively affect CRF [62]. The lack of impact in MSF mediation potentially could be the effect of a lack of favorable changes in muscle mass. Therefore, it is suggested to respect sex differentiation in applying training loads during the HIIT intervention. HIIT is an effective method in increasing muscle mass, even among obese individuals. However, to achieve this effect, the proper load must be inflicted [63]. Generally, males are more susceptible to building muscle mass than women in response to training loads [64]. However, our study sample was young adolescents before full maturation, and therefore, it was a common effect on MSF. The differences in MSF effect between boys and girls may be due to differences in physical fitness, whereas males are generally stronger than women, which are more flexible than men [65]. In the study by Cvetković et al. [36], HIIT showed positive effects of HIIT on CRF, and MSF expressed as change of direction speed and low impact in lower extremity power. Abovementioned observation suggests considering other MSF components to boys and girls.

## 5. Conclusions

Our results confirmed HIIT impact on CRF represented here by the Harvard step-test results among boys and girls. The synthetic variable representing musculoskeletal fitness as a composite-MSFI did not contribute valuable information. There were no premises for using such synthetic measures for boys and girls based on the same MSF components. From MSF components, only abdomen muscle strength and flexibility mediated the relationship between HIIT and cardiorespiratory fitness in the whole group of adolescents. Detailed analysis revealed a moderation effect of the sex factor, which affected mediation models. Therefore, our findings suggested the relationship between variables called by Baron and Kenny [32]—moderated mediation. It manifested the presence of mediation effects in girls but the absence of such relation in boys.

Abdomen muscle strength and flexibility seemed to significantly mediate the relationship between HIIT and CRF in the girls' group. The intervention significantly impacted abdomen muscle strength and flexibility in girls, which implied an improvement in their level of cardiorespiratory fitness. Detailed analysis indicated complete mediation of the flexibility (accounted for 36%) but only partial mediation of the abdomen muscle strength (accounted for 18%). It meant there were other confounders independently and simultaneously affecting cardiorespiratory fitness. Therefore, further work is needed to identify confounders affecting CRF. Our results could be the tip for teachers, coaches, physiotherapists, and all supervisors of the persons taking up physical activity that stimulation of the core muscles (back, abdominals, pelvis) could be effective and supportive for improving cardiorespiratory functions. Interventions for gaining CRF among adolescent girls should focus on improving both their abdomen muscle strength and flexibility. Further studies should focus on confounders of the CRF in the boys' group. It needs to consider applying other training loads to boys and girls.

Our research has shown that HIIT implemented into physical education classes, adequately supervised, and effectively improved CRF in healthy adolescents. In addition, some MSF components are engaged, which supports the CRF development as feedback. This study has identified a feasible and efficacious approach for achieving at the same time improvement in CFR and MSF among adolescent girls.

## 6. Limitations

One limitation of this work arises from a specific group—healthy adolescents with BMI in the norm and normotensive. Further researches for underweighted or overweighed persons, as well as for hypertensive ones, are needed. The second limitation relates to unequal sex distribution of the sample, in which there was a slight bias toward the female. In addition, we did not directly measure VO_2max_ but estimated CRF through physical fitness index, calculated in Harvard step-test, which has some limitations and assess CRF not very precisely. Future studies should confirm the findings with directly measured VO_2max_. Despite these limitations, this study had many methodological strengths. After finishing a project, adolescents from the control group entered an intervention (in the new school year). The intervention was conducted in typical schoolwork conditions, during specific physical education classes. Almost all students from the class were introduced to the project.

## Figures and Tables

**Figure 1:** Hypothesized moderation model of potential effects of sex (moderator) on the relationship between HIIT and CRF through MSF (mediator). Numbers indicate effects of moderation on mediation model's elements: (1) indirect influence of HIIT on CRF, (2) component: HIIT effect on MSF (MSFI, HG, ABS, FL, VJ), and (3) component: MSF (MSFI, HG, ABS, FL, VJ) effect on CRF.

**Table 1:** Descriptive statistics of the baseline measured variables and residual changes (RC) in groups.

Group	Boys		Girls	
	Intervention	Control	Intervention	Control
Variable	Mean (±sd) 95% CI	Mean (±sd) 95% CI	Mean (±sd) 95% CI	Mean (±sd) 95% CI
	RC mean 95% CI	RC mean 95% CI	RC mean 95% CI	RC mean 95% CI
Body height (cm)	176.09 (6.54)	177.63 (5.84)	164.79 (6.04)	163.99 (7.27)
	173.5-178.68	174.72-180.53	162.7805-166.81	161.66-166.31
	0.2	0.16	0.14	0.19
	0.13-0.26	0.09-0.22	0.1032-0.18	0.13-0.25

Body weight (kg)	63.74 (12.15)	64.68 (8.72)	56.35 (7.61)	56.76 (12.52)
	58.93-68.55	60.35-69.02	53.81-58.89	52.75-60.77
	-1.61	1.28	0.13	0.34
	-5.46-2.23	0.27-2.3	-0.37-0.63	-0.13-0.81

BMI (kg/m^2^)	20.51 (3.44)	20.48 (2.43)	20.69 (1.94)	21 (3.66)
	19.15-21.87	19.27-21.69	20.04-21.33	19.83-22.17
	-0.19	-0.11	0.04	0.12
	-0.5-0.11	-0.49-0.28	-0.14-0.21	-0.06-0.3

CRF (FI) (pts)	44.98 (4)	44.06 (3.46)	43.33 (4.93) 41.68	45.53 (3.4)
	43.4-46.57	42.33-45.78	- 44.97	44.44-46.62
	3.41	1.1	2.89	0.6
	1.5-5.32	-0.26-2.46	1.8-3.97	-0.45-1.66

Hand grip (kg)	45.22 (8.09)	42.83 (7.14)	31.27 (4.28)	31.83 (6.31)
	42.02-48.42	39.28-46.38	29.84-32.7	29.81-33.84
	1.02	2.25	1.12	2.03
	0.08-1.96	-0.68-5.17	0.31-1.94	1.05-3.01

Sit-ups (*n*)	26.44 (3.19)	26.94 (3.1)	19.27 (4.76)	20.6 (3.62)
	25.18-27.71	25.4-28.48	17.68-20.86	19.44-21.76
	5.17	6.39	0.85	-1.43
	3.91-6.42	2.95-9.83	-0.18-1.88	-2.32--0.55

Sit-and-reach (cm)	21.78 (7.85)	25.72 (8.37)	27.28 (6.19)	27.63 (8.18)
	18.67-24.88	21.56-29.88	25.22-29.35	25.01-30.24
	3.21	4.23	3.43	-0.76
	1.94-4.48	2.13-6.33	2.53-4.32	-2.59-1.07

Vertical jump (cm)	58.63 (8.66)	56.72 (7.5)	41.41 (6.71)	43.2 (5.89)
	55.2-62.06	52.99-60.45	39.17-43.64	41.32-45.08
	-4.66	-1.88	-0.45	-0.03
	-6.86--2.46	-4.82-1.07	-2.21-1.3	-1.59-1.52

MSFI (composite)	0.33 (0.05)	0.28 (0.07)	0.46 (0.09)	0.42 (0.08)
	0.31-0.35	0.24-0.31	0.44-0.49	0.4-0.45

It did not calculate residual changes for MSFI (MSFI is based on residual changes for each motor test–as a component).

**Table 2:** Moderation effects of sex on the three elements of mediation models (1-3 on Figure 1) in the relationship between HIIT and CRF through MSF (MSFI, HG, ABS, FL, VJ)—*p* values.

Mediator	Indirect effect	Components	
	HIIT⇨CRF (1)	HIIT⇨MSF (2)	MSF⇨CRF (3)
MSFI	0.884	0.843	0.704
HG	0.988	0.881	0.980
ABS	0.822	0.011	<0.001
FL	0.638	0.001	0.004
VJ	0.851	0.265	0.179

**Table 3:** Indirect effects—*p* values.

Indirect effect	Average	Boys	Girls
MSFI	0.442	0.288	0.645
HG	0.544	0.563	0.576
ABS	0.771	0.253	0.031
FL	0.801	0.497	0.024
VJ	0.816	0.357	0.731

**Table 4:** Mediation effects: direct and components (in the model).

Test	Effect	*B*	SE	95% CI	*Z*	*p*
ABS	Direct	2.974	0.762	1.481–4.467	3.90	0.001
	Components:					
	HIIT⇒ABS	2.283	0.659	0.990–3.575	3.460	<0.001
	ABS⇒CRF	0.303	0.122	0.063–-0.543	2.470	0.013

FL	Direct	1.462	0.782	-0.071	2.995	0.062
	Components:					
	HIIT⇒ABS	4.181	1.019	2.185 6.178	4.100	<0.001
	ABS⇒CRF	0.196	0.079	0.041–0.352	2.480	0.013

*B*: estimate regression; SE: standard error of the regression; CI: confidence coefficient index; HIIT: high-intensity interval training; CRF: cardiorespiratory fitness; ABS: sit-ups test; FL: sit-and-reach test.

## Data Availability

Data are available upon request due to ethical restrictions regarding participant privacy. Requests for the data may be sent to the corresponding author.
